# Effects of Ganoderic Acid A on Gastrointestinal Motility and Brain-Gut Peptide in Rats with Functional Dyspepsia

**DOI:** 10.1155/2022/2298665

**Published:** 2022-05-31

**Authors:** Wei Yang, Rui Liu, LinHua Zhou, Xiao Chen, YanYan Hu

**Affiliations:** ^1^Department of Gastroenterology, Xiangyang Central Hospital, Affiliated Hospital of Hubei University of Arts and Science, Xiangyang, Hubei Province 441021, China; ^2^Medical School of Xiangyang Vocational and Technical College, Xiangyang, Hubei Province 441022, China; ^3^School of Cosmetology, Yichun University, Yichun, Jiangxi Province 336000, China; ^4^School of Nursing, Yichun Vocational Technical College, Yichun, Jiangxi Province 336028, China

## Abstract

**Objective:**

The therapeutic effect of drugs for functional dyspepsia (FD) is still limited. Ganoderic acid A (GAA) has anti-inflammatory and cellular protective activities. The aim of this study is to explore the therapeutic effect of GAA on FD.

**Methods:**

The FD rat model was established via tail damping and forced exercise fatigue. The gastric emptying rate and intestinal propulsion rate of the rats in each group were then detected, and the pathological damage of gastric antrum and duodenum tissues was observed by hematoxylin-eosin (HE) staining. An enzyme-linked immunosorbent assay (ELISA) was conducted to determine the levels of motilin (MTL), vasoactive intestinal peptide (VIP), leptin, gastrin (GAS), calcitonin gene-related peptide (CGRP), and somatostatin (SS) in plasma, and Western blot was used to detect the protein expression levels of occludin, zonula occluden-1 (ZO-1), and junctional adhesion molecule-1 (JAM-1) in the duodenal tissue.

**Results:**

Treatment with GAA significantly raised the gastric emptying rate and intestinal propulsion rate of FD rats and histologically alleviated the gastric and duodenal damage. Meanwhile, GAA positively regulated the secretion of brain-gut proteins, such as upregulation of MTL, GAS, and SS and downregulation of VIP, leptin, and CGRP. In addition, GAA treatment increased the protein expression levels of occludin, ZO-1, and JAM-1 in the duodenal tissue of the FD rats.

**Conclusion:**

GAA may exhibit protective effects on FD by regulating the secretion of brain-gut peptide, protecting the intestinal barrier and improving gastrointestinal motility.

## 1. Introduction

Functional dyspepsia (FD), also known as nonulcer dyspepsia, is one of the most common functional gastrointestinal disorders. FD is usually characterized by epigastric pain, persistent and recurring epigastric bloating, early satiety, anorexia, nausea, and abdominal discomfort, etc. [1]. It is reported that the prevalence of FD varies greatly among different regions, such as 10–40% in Western countries but 5–30% in Asia [2]. Risk factors for FD include gastrointestinal infection and diarrhea, gastric emptying, impaired gastric regulation, duodenal inflammation, mucosal permeability, use of antibiotics or anti-inflammatory drugs, early environmental microbial exposure, and psychosocial factors. And some lifestyle factors are also covered, such as smoking, obesity, stress, and psychosocial status. [3–5]. Studies have shown that patients with FD, without timely treatment, are at risk of developing peptic ulcer and gastric cancer, which will result in a higher cost of treatment for the condition [6–8]. At present, the clinical treatment methods for the symptoms of FD mainly include dietary adjustment, drug treatment, and psychological treatment. The approach of adjusting dietaries takes a relatively long time and is still under investigation. Compared with psychological treatment, which usually plays an auxiliary role in FD treatment, response to drug treatment may occur relatively quickly. However, most drugs applied to clinical studies have limited improvement in symptoms [9, 10]. Therefore, it is crucial to find new and effective drugs for treating FD.

*Ganoderma lucidum* (*G*. *lucidum*) is a large white-rot fungus which belongs to basidiomycete. It has an applicative history of 2000 years in China and other Asian countries and has been regarded as a beneficial food to the body all the time [11]. With the deepening of research, it has been found that *G*. *lucidum* has the potential to treat diseases. The root bark, mycelium, and spores of *G*. *lucidum* contain about 400 different biological active compounds, mainly including triterpenoids, polysaccharides, nucleotides, sterols, steroids, fatty acids, proteins/peptides, trace elements, and other substances [12]. These compounds possess various activities, such as immunomodulation, anti-inflammation, analgesia, antitumor, sleep promotion, antibacterial, antivirus, hypolipidemia, antioxidation, and free radical scavenging [13]. And studies have shown that *G*. *lucidum* pills can promote the healing of chronic gastric ulcers induced by ethanol and significantly improve gastric mucosal injury [14]. Triterpenoids are the most promising candidates for clinical drugs whose natural compounds have pharmacological activities [15]. Ganoderic acid A (GAA), as the most important component of triterpenoids, has relatively good anti-inflammatory, antitumor, and other pharmacological activities. Das et al. found that GAA inhibited the growth of grade III meningioma cells by changing the protein expression of p-AKT, p-mTOR, and Wnt-2 [16]. Studies conducted by Chi et al. showed that GAA may decrease lipopolysaccharide (LPS)-induced IL-1*β*, IL-6, and TNF-*α* release from mouse-derived cortical microglial cells when inhibiting the expression of nuclear factor (NF)-*κ*B (p65) [17]. However, little is known about the effect of GAA on FD. Therefore, in this study, the FD rat model was established and GAA treatment was administered to the animals to observe its therapeutic effect on FD. The pathological damage of gastrointestinal tissue was assessed and the levels of various brain-gut peptides and the expression of tight junction (TJ)-associated proteins were determined in the rats mainly via hematoxylin-eosin (HE) histopathological staining, enzyme-linked immunosorbent assay (ELISA), and Western blot. And domperidone (Dom) was used as a positive control for FD rats. This evidence may contribute to the development of a new drug and provides proof for the relief of FD symptoms.

## 2. Materials and Methods

### 2.1. Construction and Grouping of the FD Rat Model

This study was approved by the Ethics Committee of Xiangyang Central Hospital (C202205-8), and the relevant experiments were carried out in accordance with the approved guidelines. Domperidone maleate (Dom, a dopamine antagonist) was purchased from Janssen Pharmaceutical Co., Ltd. (Xi'an, Shaanxi, China). GAA was obtained from Med ChemExpress (Shanghai, China). Following the method of Liang et al. [18], the FD model was established by stimulating semistarved rats via tail damping, provocation, and forced exercise fatigue, four times a day for 10 consecutive days. Each time, a gauze-wrapped hemostat was used to clamp the distal third of the rat's tail for 30 min without skin damage. Afterwards, the rats were required to run for 10 min for exercise fatigue, four times a day for 10 consecutive days.

A total of 24 adult male SD rats weighing 180–220 g were selected and randomly divided into four groups: the control group, the FD model group, the GAA-treated FD model group, and the DOM-treated FD model group. Rats in the control group received a normal diet and an equal volume of normal saline (NS) via intragastric administration every day. The other rats were induced FD and 10 days later, they received an equal volume of NS, 40 mg/kg GAA, or 3 mg/kg domperidone (Dom) through stomach perfusion every day for four weeks, respectively. After the last gavage, the rats in each group were fasted for 24 h. On the next day, three rats in each group were randomly selected for abdominal aorta blood sampling under anesthesia.

### 2.2. Detection of Gastric Emptying and Intestinal Propulsion

Rats in each group were fed with nutritional semisolid paste (2 mL) by gavage and euthanized after 30 min. The abdominal cavity was then opened to ligate the cardia and pylorus of the stomach, followed by excision of the entire stomach and small intestine. The whole stomach was weighed to get *W*1. After removing the gastric contents, the stomach was dried with a filter paper and the dry weight (*W*2) was measured with the weight of the nutritional semisolid paste recorded (*W*3). The gastric emptying of rats in each group was calculated using the following formula: gastric emptying = (*W*1 − *W*2)/*W*3 × 100%, and the intestinal propulsion rate was calculated as well by using the following formula: intestinal propulsion rate = L2 (the distance semisolid paste travels from the pylorus)/L1 (full length of the small intestine from the pylorus to the ileocecal junction) × 100%.

### 2.3. HE Staining

The rat gastric and duodenal tissues were fixed in a fixative, embedded in paraffin, and cut into sections. The sections were stained according to the instructions of the HE staining solution and observed and photographed under a microscope.

### 2.4. ELISA Assay

The blood sample was allowed to stand for 30 min and then centrifuged at 4°C at 2000 r/min for 20 min. The supernatant was collected into new centrifuge tubes and stored in a −80°C refrigerator. The serum levels of motilin (MTL), vasoactive intestinal peptide (VIP), leptin, gastrin (GAS), calcitonin gene-related peptide (CGRP), and somatostatin (SS) were detected in accordance with the instructions of the corresponding ELISA detection kit (Jiancheng Bioengineering, Nanjing, Jiangsu, China). The absorbance value at 450 nm was also detected.

### 2.5. Western Blot

The rat duodenal tissues were lysed with radio-immunoprecipitation assay (RIPA) lysis solution (Solebo Life Science, Beijing, China) and centrifuged at 12000 rpm/min at 4°C for 30 min to obtain the supernatant lysate. 20 *μ*g of protein of the lysate was separated through sodium dodecyl sulfate-polyacrylamide gel electrophoresis (SDS-PAGE), transferred on a polyvinylidene fluoride (PVDF) membrane, blocked in 5% nonfat dry milk for 1-2 h, and incubated with the primary antibodies (occludin, zonula occluden-1 (ZO-1), JAM-1, *β*-actin; all from Abcam (Cambridge, United Kingdom)) overnight at 4°C and secondary antibodies (Abcam) at room temperature for 1 h. The membrane was rinsed before and after the secondary antibody incubation. Subsequently, the sample was developed with electrochemiluminescence (ECL) (Beyotime, Shanghai, China) and then photographed under a gel imaging system. With *β*-actin as the internal reference, Image J software was used to analyze the gray level of protein bands.

### 2.6. Statistical Analysis

All results were analyzed by SPSS 26.0 (IBM-SPSS, Chicago, IL, USA) software and expressed as mean ± standard deviation (SD). One-way ANOVA analysis of variance and independent sample *t-*test analysis were used for analyzing the difference between groups. *p* < 0.05 indicates significant differences.

## 3. Results

### 3.1. Effect of GAA on Gastric Emptying and Intestinal Propulsion in FD Rats

To investigate the impact of GAA on gastrointestinal motility in FD, we established a FD rat model and assessed the condition of gastric emptying as well as intestinal propulsion. The results showed that compared with the control group, the FD model group had significantly decreased gastric emptying rate and intestinal propulsion rate (*p* < 0.01), suggesting that the FD rat model was successfully established in this study. Then, FD rats were intragastrically administered with 40 mg/kg GAA and 3 mg/kg Dom (positive drug), respectively. As a sequence, the gastric emptying rate and intestinal propulsion rate of the GAA group and Dom group were significantly higher than those of the FD group (*p* < 0.01) with GAA exhibiting a greater therapeutic effect (Figures 1(a) and 1(b)). These evidence suggests that GAA may increase the gastric emptying rate and intestinal propulsion rate in FD rats.

### 3.2. Protective Effect of GAA on the Pathological Injury to Gastric and Duodenal Tissue in FD Rats

Subsequently, we collected the gastric and duodenal tissues of the rats in each group and performed HE staining to evaluate the histopathological damage. Compared to thinning, rupture, and basal layer congestion of gastric mucosa in the gastric and duodenal tissues of the FD group, the tissues in the GAA and Dom groups revealed intact gastric structure (Figure 2(a)). In addition, epithelial cell swelling, focal necrosis, exfoliation, and massive inflammatory cell infiltration were seen in the duodenal tissue sections of the FD group. Upon treatment with GAA or Dom, however, these symptoms almost disappeared and only mild hyperemia and inflammatory cell infiltration remained with intact duodenal mucosa (Figure 2(b)). Collectively, GAA could significantly alleviate the gastric and duodenal tissue injury in FD rats.

### 3.3. GAA Affects the Level of Brain-Gut Peptide in Serum of FD Rats

Previous studies have depicted the important role of bidirectional interaction between the brain and gut in FD patients as MTL, GAS, leptin, VIP, SS, CGRP, and other brain-gut peptides are transported into this cycle of bidirectional interaction [19, 20]. Herein, we checked the levels of those brain-gut peptides in the serum of the rats in each group using ELISA. The results showed that compared with the control group, the serum levels of MTL, GAS, and SS in rats of the FD group were significantly decreased, while VIP, leptin, and CGRP increased. Of note, GAA treatment greatly restored the levels of MTL, GAS, and SS in FD rats and reduced contents of VIP, leptin, and CGRP, exhibiting similar effect on brain-gut peptide as Dom with no significant difference (Figures 3(a)–3(f)). It is suggested that GAA may restore the level of brain-gut peptide in the serum of FD rats.

### 3.4. GAA Improves the Barrier-Function Damage of Duodenal Mucosa in FD Rats

Furthermore, we observed that duodenal mucosal integrity was impaired in FD rats which led to symptoms of FD, so we investigated whether GAA could restore duodenal mucosal function by regulating TJ proteins (occludin, ZO-1, and JAM-1). As revealed by Western blot, the protein expression levels of occludin, ZO-1, and JAM-1 in the duodenal tissue of the FD rats declined significantly (*p* < 0.01), indicating impaired intestinal barrier function. Importantly, these protein levels were significantly restored evidently in the presence of GAA (*p* < 0.05) (Figures 4(a) and 4(b)), suggesting that GAA may improve the impaired barrier-function of duodenal mucosa in FD rats.

## 4. Discussion

FD is a disease affecting many facets of patients' life [21], mainly including postprandial fullness, early satiety, or/and physical discomfort such as epigastric pain or burning sensation, as well as the cost of time and economy [22]. Gastric emptying disorder is considered to be the physiological mechanism of FD, but presently, no good prokinetic drugs can effectively treat such condition [9]. In this study, the FD rat model was established through tail damping, forced exercise, and other processes. It was found in the experiments that the rates of gastric emptying and intestinal propulsion in FD rats were significantly lower than those in normal rats. Moreover, the pathological damage appeared in the gastric and duodenal tissues of FD rats. These indicators of the FD model rats confirmed that the FD rat mode was successfully established. In addition, FD patients are often accompanied with psychiatric comorbidities. Some studies thereby paid attention to the therapeutic effects of central nervous system modulators on early satiety and nausea in FD patients with depression or anxiety comorbidities [23]. However, most psychotropic drugs are accompanied with certain side effects and should be used with care. In addition, the application of Chinese herbal medicine in FD has also received increasing attention, and the herbal combination preparation STW5 is one of the most studied compounds. It is composed of various Chinese herbs, such as angelica root, milk thistle fruit, coriander fruit, celandine balsam leaf, and mint leaf. Clinical data showed that STW5 relieved gastrointestinal symptoms without adverse side effects [24], suggesting that Chinese herbal ingredients may have better efficacy in FD. In this study, we found that administration of GAA significantly improved gastric emptying and intestinal propulsion in FD rats and alleviated gastric and duodenal injuries. Although there is currently no research relating to the function of GAA in FD, multiple studies have noted the protective role of GAA in various cellular or tissue injuries. For example, Wan et al. found that GAA can alleviate LPS-induced lung tissue damage [25]. Li et al. noted that GAA may ameliorate hypoxia-induced PC12 cell damage [26]. Therefore, it is suggested that GAA has the function of treating FD symptoms and has the potential to become a drug for the treatment of this disease.

Communication between the central and enteric nervous systems is indispensable to the links sustaining life activities. And peptides such as brain-gut peptides, distributed in both the gastrointestinal and nervous systems, act as messengers during this process. It is reported that FD patients with delayed gastric emptying had lower levels of SS, MTL, and GAS with elevation of VIP, leptin, and CGRP levels [19]. Among these proteins, during the fasting state, MTL is released from *M* cells located in the proximal duodenum and acts as a stimulus to gastric antrum contraction, thereby exerting the function of signaling starvation [27]. SS is released in both the stomach and small intestine and has a strong inhibitory effect on gastrointestinal motility and secretion [28]. GAS is the main stimulator of gastric acid secretion, released by *G* cells in the stomach. These brain-gut peptides are all biomarkers reflecting the function of the gastrointestinal tract. Consistent with the results shown in the study of Liang et al. [18], we also found that the serum levels of MTL, GAS, and SS in FD rats were significantly decreased, while the levels of VIP, leptin, and CGRP increased. Moreover, administration of GAA restored the levels of MTL, GAS, SS, VIP, leptin, and CGRP, and its therapeutic effect was not significantly different from Dom treatment, indicating that GAA has the function of improving FD symptoms. And, the study of Jonsson et al. found that the number of duodenal endocrine cells in FD patients was significantly decreased, leading to an impairment of mucosal barrier function [29]. When dysfunction occurs to the mucosal barrier, immune response would be elicited by pathogens or allergens, which crosses the intestinal epithelium of the duodenum. Furthermore, this localized response may trigger intestinal barrier damage, extraintestinal symptoms, and even a systemic immune response [30]. It is noted that there are significant correlations between mucosal permeability and TJ protein expression in ulcerative colitis and irritable bowel syndrome [31, 32]. As an important part of the epithelial mechanical barrier, TJ proteins, such as occludin, ZO-1, and JAM-1, play an important role in protecting the intestinal mucosa from foreign antigens, toxins, and environmental microorganisms [33]. We found that the levels of occludin, ZO-1, and JAM-1 in the duodenal tissue of FD rats were significantly decreased and their levels were significantly restored upon GAA treatment. It is suggested that GAA may protect gut function by promoting the expression of TJ protein, thereby avoiding further damage to the gut.

At present, quite a few studies have explored the mechanism underlying GAA in various diseases. For example, Wang et al. found that GAA contributes to inflammation and lipid deposition through the Notch1/PPAR*γ*/CD36 signaling pathway [34]. Bao et al. found that GAA exerts neuroimmune and antidepressant effects by regulating FXR, a receptor of bile acid [35]. Zhang et al. found that GAA plays a protective role in H9c2 cardiomyocytes of hypoxic injury via up-regulation of miR-182-5p [36]. To sum up, GAA may play its role through molecular signaling pathways, receptors, miRNAs, etc. This study has mainly explored the function of GAA in FD but failed to fully reveal the mechanism of action of GAA. Therefore, further experiments and exploration are expected to provide the clinical application of GAA with more functional experimental basis and mechanism action theories.

## 5. Conclusion

Collectively, GAA may improve gastric emptying and intestinal propulsion through regulation of the secretion of brain-gut peptides to protect the intestinal barrier, thereby improving FD. This evidence highlights the potential of GAA to be a promising therapeutic drug for FD.

## Figures and Tables

**Figure 1:** GAA improves gastric emptying and intestinal propulsion in FD rats. Effects of GAA on gastric emptying rate (a) and gastrointestinal propulsion rate (b) in the indicated groups. FD: functional dyspepsia rat model group. GAA: group of the FD rats treated with 40 mg/kg ganoderic acid A. Dom group: group of the FD rats treated with 3 mg/kg domperidone (Dom). ^*∗∗*^*p* < 0.01*vs*. control group, ^*##*^*p* < 0.01 and ^*#*^*p* < 0.01*vs*. FD group.

**Figure 2:** GAA attenuates gastric and duodenal tissue injury in FD rats. (a) HE staining was used to observe the pathological damage of gastric tissue (100 ×; Black arrows indicate disorganized tissue structure and red arrows indicate erythrocyte infiltration) and (b) duodenal tissue (100 × and 400 ×; Black arrows indicate inflammatory cell infiltration and red arrows indicate erythrocyte infiltration) of rats in the indicated groups.

**Figure 3:** GAA affects the level of brain-gut peptide in the serum of FD rats. ELISA was used to detect the levels of MTL (a), VIP (b), leptin (c), GAS (d), CGRP (e), and CGRP (f) in the serum of rats in the indicated groups. ^*∗*^*p* < 0.05 and ^*∗∗*^*p* < 0.01*vs*. control group; ^*##*^*p* < 0.01 and ^*#*^*p* < 0.01*vs*. FD group.

**Figure 4:** GAA attenuates barrier-function damage of duodenal mucosa in FD rats. (a, b) Images showing the typical Western blot (left panels) to detect the expression levels of occludin, ZO-1, and JAM-1 in the duodenal mucosa of rats in the indicated groups. The average data from three independent assays of the occludin, ZO-1, and JAM-1 in the indicated groups are presented as bar charts. ^*∗∗*^*p* < 0.01*vs*. control group; ^*#*^*p* < 0.05 and ^*##*^*p* < 0.01*vs.* FD group.

## Data Availability

The data used to support the findings of this study are available from the corresponding author upon request.
